# Charcot-Marie-Tooth Disease as a Risk Factor for Periprosthetic Fractures in Tibiotalocalcaneal Fusion With Intramedullary Nailing

This article has been retracted.

**DOI:** 10.7759/cureus.28036

**Published:** 2022-08-15

**Authors:** Ashwin Bhadresha, Baljinder S Dhinsa

**Affiliations:** 1 Trauma and Orthopaedics, William Harvey Hospital, Ashford, GBR

**Keywords:** periprosthetic fracture, hindfoot arthrodesis, tibiotalocalcaneal arthrodesis, hindfoot nailing, charcot-marie-tooth disease

## Abstract

Introduction

The treatment for severe fixed hindfoot osteoarthritis secondary to Charcot-Marie-Tooth disease (CMT) is tibiotalocalcaneal (TTC) arthrodesis. In our centre, we have noticed a disproportionate rate of periprosthetic fractures in CMT patients following TTC arthrodesis with retrograde hindfoot nailing. The aim of this study was to test this hypothesis by evaluating our local cohort of TTC arthrodesis with retrograde hindfoot nailing.

Methods

A retrospective review of patients who had TTC arthrodesis with intramedullary nailing was conducted over a seven-year period.

Results

There were 45 patients (30 male, 15 female) in our cohort. Forty-one patients achieved radiological and clinical fusion of their TTC arthrodesis. All three patients who had CMT sustained periprosthetic fracture at the tip of the nail at an average of four (range: 2.5-6) months from index operation. In comparison, no patients in the rest of the cohort sustained periprosthetic fractures. The nail position of the patients with CMT was central in both planes in all three patients. None of the patients with CMT had abutment of the cortex on either plane.

Conclusion

We found that there was a disproportionate rate of periprosthetic fractures in CMT patients in our cohort of TTC arthrodesis with retrograde hindfoot nailing. This suggests that CMT is a significant risk factor. The authors propose a longer nail to reduce the lever arm, with a long period of protected weight bearing till union, followed by consideration of elective removal of the nail to prevent this phenomenon from occurring.

## Introduction

Charcot-Marie-Tooth disease (CMT) is the most common inherited demyelinating neuropathy, affecting approximately one in 2500 people [1]. The age of presentation for CMT varies depending on the subtype, but may occur anytime from early childhood through to late adulthood. Symptoms generally fall into three categories, namely loss of sensation, muscle weakness, and bony deformity. The neuropathy and muscle weakness are often noticed first in the feet and lower limbs. The deformity develops over time and gradually becomes rigid and severe. CMT is a slow progressive disorder unlike Charcot neuroarthropathy, which is acute and is characterized by joint destruction and dislocations [2]. Alongside CMT, peripheral neuropathy can also be a manifestation of diabetes mellitus (DM) yet they affect peripheral nerve fibres of different diameters [3]. Nardone et al. noted that changes in both body sway and stance phase of gait were larger in diabetic neuropathy than in CMT1A3, the most common subtype of CMT. This indicates more impaired static and dynamic control of balance when the neuropathy affects both the small and large afferent fibres [3].

The treatment algorithm of deformity and hindfoot osteoarthritis in CMT is affected by three factors: which motor units remain functional, how flexible or rigid are the established deformities, and if ligamentous laxity is present [4]. The motor examination should focus on the relative balance of agonist-antagonist pairs that generate foot deformity. In CMT, the foot extrinsics overpower the intrinsics resulting in hallux claw toe [4]. The rigidity of the deformities determines to what degree tendon transfers, bony correction, or fusion can be used for correction, as well as the likelihood of a successful correction with bracewear [4]. Supple deformities identified with an early surgical approach can be corrected with soft-tissue surgery whereas rigid deformities need fusion and extra-articular osteotomies. Ligamentous laxity resulting in varus alignment of the hindfoot is often the first presenting complaint, and can lead to a lifetime of severe inversion injuries [4].

Although conservative measures exist as a means of therapeutic intervention as aforementioned, the foot deformities and associated neuropathy can lead to chronic ulceration and osteomyelitis, which may eventually require amputation [5]. Tibiotalocalcaneal (TTC) arthrodesis using an intramedullary (IM) nail or frame is often the only alternative to limb amputation because the deformity and osteoarthritis are severe and therefore not possible for joint preserving operations [6]. The goal of treatment is a pain-free, plantigrade, shoeable foot [7]. Although TTC arthrodesis has been shown to be an effective technique, it is not as reliable in patients with Charcot neuropathy and those with complex co-morbidities, including obesity and altered bone metabolism [8]. Perioperative and postoperative complications have been reported among this cohort for this procedure. Other complications may include non-union, malunion, and infection [5,8].

The senior author noticed a disproportionate rate of periprosthetic fractures following TTC arthrodesis with retrograde hindfoot nailing in patients with CMT disease. This observation has not been previously reported in the literature to the authors’ knowledge. This study was therefore undertaken to test this hypothesis by comparing them to our local cohort of TTC arthrodesis with retrograde hindfoot nailing.

This study was previously presented as a meeting abstract poster presentation at the Association of Surgeons in Training International Virtual Surgical Conference on March 5, 2021. 

## Materials and methods

Patients who had a retrograde hindfoot nail were identified using our local database. Patients requiring a retrograde hindfoot nail for traumatic osteoporotic ankle fractures and revision cases were excluded from the study. All patients had radiological evidence of severe arthritis of the ankle and subtalar joints, and had failed appropriate conservative treatment. The operations were carried out by two fellowship-trained foot and ankle consultants. The selected sample group consisted of 45 patients (30 men and 15 women) who underwent elective TTC arthrodesis for osteoarthritis between September 2010 and June 2017. Four patients were deceased at the time of the study. The study was conducted at the Royal Gwent Hospital, Newport, Wales.

Clinical records were retrospectively reviewed for this cohort of patients and complications were recorded. Radiographs were also reviewed. The long axial view was used to measure hindfoot alignment preoperatively and postoperatively to assess the magnitude of varus and valgus deformity and its correction [9]. The radiological degree of long axial hindfoot alignment was defined as the angle between the mid-diaphyseal axis of the tibia and the calcaneus axis [9]. Postoperative anteroposterior and lateral radiographs were used to evaluate the nail position in the tibial canal. We defined union of the arthrodesis joint as the time when the patient reported no bony pain, warmth, and swelling over the fusion site or only mild activity-related discomfort and there was radiographic evidence of healing with bridging trabeculae of at least 75% of the cross-section on both views. All radiographs were evaluated by two surgeons, each of whom was blinded to all other patient data. Delayed union was defined as a lack of clinical and radiological evidence of union, bony continuity or bone reaction at the arthrodesis site if three months have elapsed from the initial operation. Non-union was defined as no radiological evidence of union of arthrodesis site after nine months, following serial radiographs. When indicated, CT was performed to assess for union and was evaluated by independent radiologists.

TTC arthrodesis was performed using the Valor Hindfoot Fusion System (Wright Medical, Tennessee, United States) in the majority of patients (64%). The Phoenix Ankle Arthrodesis Nail System (Biomet, Warsaw, United States) was used in the rest. This was due to surgeon preference. The Valor and Phoenix hindfoot nail are both straight nails with an internal compression system. The nail diameter was 10 mm in 28 patients, 11 mm in 11 patients, 11.5 mm in one patient and 12 mm in two patients. The length of the nail was 150 mm in 42 patients, 180 mm in one patient, 200mm in one patient and 210 mm in one patient.

Surgical technique

The patient was placed in a supine position and the ankle was placed in neutral dorsiflexion. A lateral transfibular approach was used in all patients. A guide wire was then introduced under fluoroscopic control down the centre of the calcaneus, talus, and tibial medullary canal. The opening reamer was then advanced over this wire to the distal tibial physeal scar. A ball-tipped guide wire was placed into the tract and was followed by sequential reaming with flexible reamers until 1-1.5 mm greater than the nail diameter was achieved. After nail insertion, two interlocking screws were placed proximally in the tibia, with at least one interlocking screw placed through the calcaneus. Compression of the fusion sites was obtained with the internal device of the nail. In 29 patients (64%), bone graft was used. This consisted of DBX demineralized bone matrix (MTF Biologics, New Jersey, United States): an allograft bone void filler. Fibula excision was undertaken in 30 patients (67%), and the medial malleolus was excised in 16 patients (30%). 

Post-operative protocol

The patients were put into a below-knee backslab for the first week. The wound was checked at the end of week one and the patients were converted into a full below-knee polymer cast and were allowed to touch weight-bear on it. The patients were followed up at six weeks with the removal of polymer cast and radiographs. If the radiographs were satisfactory and there was no pain on stressing the fusion sites, they were allowed to gradually weight-bear as comfortable in an aircast walker and wean off as able. All patients were referred to physiotherapy for gait instruction. They were followed up further at three months, six months, and one year with radiographs on arrival.

Statistical analyses

Statistical analysis of recorded parameters between both groups was performed with Student's t-test for parametric values, Mann-Whitney U test for non-parametric values whilst Fisher's exact test or Chi-square test was used for categorical data. Fisher's exact test was used in proportion comparisons where values in any cells fell below five. Chi-square test was used in proportion comparisons where values in all cells were above five. Significance was defined as p≤0.05. Data were analyzed using IBM SPSS Statistics for Windows, Version 20.0 (Released 2011; IBM Corp., Armonk, New York, United States).

## Results

Demographics

The average age at the time of operation in our cohort was 63 years (range: 44-87 years). There were 30 males and 15 females. Twenty-one patients (47%) underwent arthrodesis on the left side. Sixteen patients (36%) were smokers, five patients (11%) were diabetic, and six patients (13%) had rheumatoid arthritis. Of the five diabetic patients, one had a previous Charcot arthropathy while the rest had no neuropathy. Five patients in the non-CMT group had diabetes whilst no patients in the CMT group had diabetes. Out of the 45 patients in our cohort, three had CMT disease (7%). Table 1 describes the patient demographics of the study population between CMT patients and the rest of the cohort. There was no statistical significance between the age, sex, BMI, and smoking status of both cohorts. The average follow-up was 48 months (range: 13-87). In terms of pre-operative deformity, all CMT patients had a varus deformity. The mean varus deformity in this cohort was seven degrees measured radiographically. A further breakdown is available in Table 1. 

**Table 1:** Demographics of patients with CMT compared to the rest of the study population CMT: Charcot-Marie-Tooth disease

Patient demographics		
Parameters	CMT	Non-CMT
Gender, n		
Male	2	28
Female	1	14
Mean age, years (range)	57 (53-60)	64 (44-87)
Mean body mass index, kg/m^2 ^(range)	30 (29-30)	32 (19-50)
Fused side, n		
Left	3	18
Right	0	24
Co-morbidities, n		
Smoking	2	14
Diabetes	0	5
Rheumatoid arthritis	0	6
Pre-operative deformity, n		
Valgus	0	8
Varus	3	16
Equinus	0	2

Clinical outcome

Forty-one patients (91%) in our cohort achieved radiological and clinical union. Table 2 compares the treatment outcomes of CMT patients to the rest of the patients who underwent hindfoot nailing. The four nonunions were in the non-CMT cohort and had revision surgery. The patient who had a previous Charcot arthropathy, unfortunately, ended up with an infected nonunion and had a below-knee amputation. There were two superficial infections, which were successfully treated with antibiotics. There were six nerve paraesthesias in the non-CMT cohort and none in the CMT cohort but the longstanding neuropathy in the CMT cohort could have skewed this finding. A significant finding was that all three patients with CMT sustained periprosthetic fractures. In comparison, no patients in the rest of the cohort sustained periprosthetic fractures.

**Table 2:** Treatment outcomes of patients with CMT compared to the rest of the study population CMT: Charcot-Marie-Tooth disease

Outcome of Treatment		
Outcome of Treatment	CMT	Non-CMT
	n	n
	3	42
Mean follow-up (months)	25.6 (range 19-40)	49.7 (range: 13-87)
Radiological fusion	3	38
Time to union (weeks)	8 (6-10)	8 (6-12)
Non-union	0	4
Nerve paraesthesia	0	6
Periprosthetic fracture	3	0
Deep infection	0	1
Superficial infection	0	2
Metalwork failure	0	3
Deep vein thrombosis	0	1
Re-operation	3	6

Radiological analyses

Table 3 shows the postoperative radiographic analysis of the nail position. The nail position of the patients with CMT was central in both planes in all three patients. None of the patients with CMT had abutment of the cortex on either plane. This compares more favourably with the non-CMT group in terms of nail position. All three CMT patients had a 150 mm x 10 mm nail, which was the smallest possible length and diameter. In two patients, the operation notes documented that the intramedullary canal was very tight.

**Table 3:** Position of nail radiologically of patients with CMT compared to the rest of the study population AP: anteroposterior; CMT: Charcot-Marie-Tooth disease

Position of nail				
		CMT	Non-CMT	p-value
AP radiograph	Central	3	32	1.000
	Medial	0	4	
	Lateral	0	7	
Lateral radiograph	Central	3	24	0.728
	Anterior	0	11	
	Posterior	0	7	
	Abutment of cortex on either view	0	9	1.000

The three CMT patients who sustained periprosthetic fractures had bilateral CMT with severe fixed Cavovarus hindfoot osteoarthritis, and in all three cases, it was the worst side that was operated on first.

Case One

Case one was a 59-year-old gentleman at the time of operation (Figures 1a, 1b). He had an uneventful recovery (Figures 1c, 1d). He sustained a periprosthetic fracture when he lightly knocked his leg against a worktable (Figures 1e, 2a) at six months after surgery and presented to the Emergency Department because of mild pain. This occurred on two occasions and he was treated conservatively with a Sarmiento walking cast as the fracture was undisplaced (Figures 2b, 2c). The CT scan after the second periprosthetic fracture confirmed union of the fracture site at eight weeks from the second incident, and the nail was electively removed (Figures 2d, 2e).

**Figure 1:** Radiological images of Case 1. (a) and (b): Preoperative AP and lateral radiographs of a 59-year-old gentleman with severe Cavovarus osteoarthritis secondary to Charcot-Marie-Tooth disease; (c) and (d): Postoperative AP and lateral radiographs showing that the alignment of the hindfoot nail being centre-centre on both views; (e) AP radiograph showing a periprosthetic fracture when he lightly knocked his leg against a worktable AP: anteroposterior

**Figure 2:** Radiological images of Case 1. (a) lateral radiograph showing a periprosthetic fracture when he lightly knocked his leg against a worktable; (b) and (c): AP and lateral radiographs showing a further periprosthetic fracture over healing callus; (d) and (e): AP and lateral radiographs following elective nail removal AP: anteroposterior Although radiographs suggest a non-union of subtalar joint, he was asymptomatic

Case Two

Case two was a 60-year-old gentleman (Figure 3 a-d) who suffered a twisting injury at two and a half months after his index operation and struggled to weight-bear (Figure 3e). He was treated with a Sarmiento walking cast as the alignment was acceptable. His intramedullary canal was extremely tight and this can be seen in his postoperative images (Figures 3c, 3d). The nail was electively removed at eight months from his index operation once CT confirmed bony union in the ankle, subtalar, and periprosthetic fracture site.

**Figure 3:** Radiological images of Case 2. (a) and (b): Preoperative AP and lateral radiographs of a 60-year-old gentleman with severe Cavovarus osteoarthritis secondary to Charcot-Marie-Tooth disease; (c) and (d) Postoperative AP and lateral radiographs showing that the alignment of the hindfoot nail being centre-centre on both views; (e) AP radiograph showing that the periprosthetic fracture after the twisting injury AP: anteroposterior

Case Three

Case three was a 53-year-old lady (Figure 4 a-d) who presented with pain and swelling three months earlier to our clinic after an uneventful post-operative recovery (Figures 4e, 5a). She denied any history of trauma. Her X-ray showed a displaced periprosthetic fracture and a decision was taken to correct this with a Taylor Spatial Frame (TSF) (Figures 5b, 5c). She fell again six months after the index operation and sustained a further periprosthetic fracture over the proximal tibia pin sites of the TSF. The proximal tibia pin sites were also complicated by infection and this was debrided and curettage. She was treated conservatively in a non-weight bearing cast with bed-to-chair transfer in hospital till union (Figures 5d, 5e). The plan is to remove her nail when she is having her second side arthrodesized.

**Figure 4:** Radiological images of Case 3. (a) and (b): Preoperative AP and lateral radiographs of a 53-year-old lady with severe Cavovarus osteoarthritis secondary to Charcot-Marie-Tooth disease; (c) and (d) Postoperative AP and lateral radiographs showing that the alignment of the hindfoot nail being centre-centre on both views; (e) AP radiograph showing a displaced periprosthetic fracture following no history of trauma AP: anteroposterior

**Figure 5:** Radiological images of Case 3. (a) Lateral radiograph showing a displaced periprosthetic fracture following no history of trauma; (b) and (c): AP and lateral radiographs showing the periprosthetic fracture treated with a Taylor Spatial Frame; (d) and (e): AP and lateral showing the healing of both periprosthetic fractures following conservative management AP: anteroposterior

## Discussion

To our knowledge, this study is the first to describe the disproportionate rate of periprosthetic fractures in CMT patients undergoing TTC fusion with intramedullary nailing. The most significant finding of this study was that all three patients with CMT sustained a periprosthetic fracture following TTC arthrodesis. By stark comparison, no patients in the local cohort of TTC arthrodesis for osteoarthritis sustained a periprosthetic fracture. The likely reason is that in patients with CMT, impaired function of the peripheral nerves results in sensory and motor neuropathy with loss of protective sensation and muscular atrophy [5,10]. This could possibly lead to repetitive micro-trauma, which causes fractures even though two of them reported trivial injury mechanisms.

The efficacy of TTC arthrodesis with an IM nail to correct severe hindfoot disease has long been documented. The present study found that 41 out of 45 patients (91%) achieved union. This high union rate with a retrograde IM nail for severe hindfoot disease has been highlighted in previous studies. Brodsky et al. reported a mean magnitude of post-operative correction to be 13.2 degrees, in addition to a high union rate and improved clinical outcomes [11]. Rammelt et al., Ettinger et al., and Taylor et al. further support these results by demonstrating that TTC arthrodesis is a viable option for the treatment of severe hindfoot disease by allowing the patient to return to a fully mobile status [12,6,13]. This may be because the IM nail provides high primary stability against rotational forces whilst also significantly reducing soft tissue damage [8]. The high union rate in our study may also be explained by the use of the internal compression mechanism in the hindfoot fusion system, which was used in all our patients [13]. Biomechanical studies have shown that systems with internal compression have demonstrated superior compressive strengths to those that rely solely on external compression [8].

Preiprosthetic fractures are a known complication following retrograde IM nailing. It may be attributable to both ankle and subtalar motion and to the difference in modulus of elasticity between bone and implant [11]. The high rate of periprosthetic fractures in this study is indeed explained by the pathophysiology of CMT as aforementioned, but it may also in part be attributed to the 150 mm nail length used in this study. Wukich et al. found that all of the tibial stress fractures sustained by diabetic patients occurred when the shortest nail (150 mm) was used [14]. A longer nail of 300 mm allows for stabilization of the nail in the isthmus of the tibial diaphysis, preventing valgus or varus toggle [14]. Similarly, Pinzur et al. found that a longer retrograde femoral nail for ankle arthrodesis decreases the risk of tibial stress fractures because all nine patients in their study achieved fusion [15]. Ankle fusion with a longer IM nailing dissipates the stress along the entire shaft of the tibia and prevents its concentration at the tip [16]. In the present study, however, the nail length was a control variable highlighting the important finding that there were no stress fractures reported in patients without CMT. In addition to the nail length, the position of the nail is also important. The position of the nail in the patients with CMT was central in both planes in all three patients. There is a greater likelihood of periprosthetic fracture if the tip of the nail is abutting one of the cortices. None of the patients with CMT had abutment of the cortex on either plane as shown in Figures 1, 2, 3, 4, 5. All three CMT had no issues with healing following their periprosthetic fractures. In fact, all three healed with abundant callus formation.

Thus far, the use of a straight retrograde IM nail for TTC arthrodesis has been evaluated; however, the high rate of periprosthetic fractures leads the clinician to question if other constructs could have better outcomes. A disadvantage of the straight IM nail is that all deformity must be corrected at the time of fixation, which can put stress on neurovascular bundles if not performed as part of a staged procedure [8]. The physiological valgus of the calcaneus with respect to the tibia means that the entry point for straight nails lies on the medial edge of the anterior process, resulting in less bony anchorage than with curved nails [12]. Budnar et al. found that the curved IM nail, therefore, had a high rate of TTC fusion with minimal plantar neurovascular complications. Its more lateral entry point addresses the anatomic danger of both the lateral plantar nerve and artery [17,18].

External fixation devices have been routinely applied for TTC arthrodesis in patients with Charcot arthropathy [15]. Pinzur demonstrated excellent results following the application of a neutrally applied three-level circular external fixator in diabetic patients affected by Charcot neuroarthropathy with midfoot deformities [19]. Dalla Paola et al. also reported an 87% fusion rate using hybrid external fixation in patients with Charcot neuroarthropathy complicated by ulcers and ankle osteomyelitis [20]. In addition, Mulligan et al. found that the lateral transfibular approach with fixed-angle plating had very similar outcomes to TTC arthrodesis with an IM nail [21]. Cadaveric studies have also shown the biomechanical superiority of a blade plate when compared to an IM nail because of its higher final rigidity and lower plastic deformation [21].

However, although these studies reported convincing results following external fixation, we do not believe it is the best construct to use for CMT patients undergoing TTC arthrodesis. Apart from their neuropathy, these patients have muscle weakness with a contralateral weak insensate deformed limb. These patients may be prone to falls after frame application, especially if the contralateral deformity is not corrected. We used the TSF as a salvage procedure for one of the periprosthetic fractures and she fell and fractured through the proximal wires (Case three). Frame arthrodesis is therefore likely to be a poor option in these patients. It is possible to use a TTC arthrodesis locking plate but the concern would be they might sustain a periprosthetic fracture at the proximal end of the plate if they fall. The best option in this group of patients is likely to be the use of a longer nail to reduce the lever arm and a long period of protected weight bearing till union, followed by consideration of elective removal of the nail. The importance of pre-operative bone density and CT scanning to assess the bone quality and other pre-operative surgical parameters in this cohort may also confer extra benefit. 

Our study had several limitations, one of which is its retrospective case-control design. We had a relatively low number of patients in the CMT cohort, but this is a relatively uncommon indication for TTC arthrodesis. Although the demographics of the patients in the two treatment groups were similar, it is possible that there were unrecognized differences between the two groups that could have affected the results. The follow-up period was significantly shorter in the CMT group, but this would not have affected the results as all three patients had periprosthetic fractures postoperatively. Another weakness of this study was there were no functional outcome measures or patient-reported outcome measures used. We only used clinical and radiological outcomes as the aim of this study was to highlight the risk of periprosthetic fracture following hindfoot nailing in CMT.

## Conclusions

In conclusion, we found that there was a disproportionate rate of periprosthetic fractures in CMT patients in our cohort of TTC arthrodesis with retrograde hindfoot nailing. This suggests that CMT is a significant risk factor. Alternative constructs include the use of a curved nail, longer nail, or external fixation. However, the authors propose a longer nail to reduce the lever arm, with a long period of protected weight bearing till union, followed by consideration of elective removal of the nail to prevent this phenomenon from occurring.
